# Prospects and applications of nanobiotechnology: a medical perspective

This article has been retracted.

**DOI:** 10.1186/1477-3155-10-31

**Published:** 2012-07-20

**Authors:** Md Fakruddin, Zakir Hossain, Hafsa Afroz

**Affiliations:** 1 Institute of Food Science and Technology (IFST), Bangladesh Council of Scientific and Industrial Research (BCSIR), Dhaka, Bangladesh; 2 Department of Microbiology, Primeasia University, Dhaka, Bangladesh

**Keywords:** Nanobiotechnology, Applications, Medical, Prospects

## Abstract

**Background:**

Nanobiotechnology is the application of nanotechnology in biological fields. Nanotechnology is a multidisciplinary field that currently recruits approach, technology and facility available in conventional as well as advanced avenues of engineering, physics, chemistry and biology.

**Method:**

A comprehensive review of the literature on the principles, limitations, challenges, improvements and applications of nanotechnology in medical science was performed.

**Results:**

Nanobiotechnology has multitude of potentials for advancing medical science thereby improving health care practices around the world. Many novel nanoparticles and nanodevices are expected to be used, with an enormous positive impact on human health. While true clinical applications of nanotechnology are still practically inexistent, a significant number of promising medical projects are in an advanced experimental stage. Implementation of nanotechnology in medicine and physiology means that mechanisms and devices are so technically designed that they can interact with sub-cellular (i.e. molecular) levels of the body with a high degree of specificity. Thus therapeutic efficacy can be achieved to maximum with minimal side effects by means of the targeted cell or tissue-specific clinical intervention.

**Conclusion:**

More detailed research and careful clinical trials are still required to introduce diverse components of nanobiotechnology in random clinical applications with success. Ethical and moral concerns also need to be addressed in parallel with the new developments.

## Introduction

Nanotechnology is a novel scientific approach that involves materials and equipments capable of manipulating physical as well as chemical properties of a substance at molecular levels. On the other hand, biotechnology uses the knowledge and techniques of biology to manipulate molecular, genetic and cellular processes to develop products and services and is used in diverse fields from medicine to agriculture. Nanobiotechnology is considered to be the unique fusion of biotechnology and nanotechnology by which classical micro-technology can be merged to a molecular biological approach in real. Through this methodology, atomic or molecular grade machines can be made by mimicking or incorporating biological systems, or by building tiny tools to study or modulate diverse properties of a biological system on molecular basis. Nanobiotechnology may, therefore, ease many avenues of life sciences by integrating cutting-edge applications of information technology & nanotechnology into contemporary biological issues. This technology has potential to remove obvious boundaries between biology, physics and chemistry to some extent, and shape up our current ideas and understanding. For this reason, many new challenges and directions may also arise in education, research & diagnostics in parallel by the extensive use of nanobiotechnology with the passage of time.

## Nanobiotechnology at a glance

Biotechnology and nanotechnology are two of the 21^st^ century’s most promising technologies. Nanotechnology (sometimes referred to as nanotech) is defined as the design, development and application of materials & devices whose least functional make up is on a nanometer scale [1,2]. Generally, nanotechnology deals with developing materials, devices, or other structures possessing at least one dimension sized from 1 to 100 nanometers. Meanwhile, Biotechnology deals with metabolic and other physiological processes of biological subjects including microorganisms. Association of these two technologies, i.e. nanobiotechnology can play a vital role in developing and implementing many useful tools in the study of life.

Nanotechnology is very diverse, ranging from extensions of conventional device physics to completely new approaches based upon molecular self-assembly, from developing new materials with dimensions on the nanoscale to investigating whether we can directly control matters on/in the atomic scale/level. This idea entails the application of fields of science as diverse as surface science, organic chemistry, molecular biology, semiconductor physics, microfabrication, etc.

## Advantages of nanobiotechnology

The pathophysiological conditions and anatomical changes of diseased or inflamed tissues can potentially trigger a great deal of scopes for the development of various targeted nanotechnological products. This development is like to be advantageous in the following ways: 1. Drug targeting can be achieved by taking advantage of the distinct pathophysiological features of diseased tissues [3]; 2. Various nanoproducts can be accumulated at higher concentrations than normal drugs [4]; 3. increased vascular permeability coupled with an impaired lymphatic drainage in tumors improve the effect of the nanosystems in the tumors or inflamed tissues through better transmission and retention [5,6]. 4. Nanosystems have capacity of selective localization in inflammed tissues [7]. 5. Nanoparticles can be effectively used to deliver/transport relevant drugs to the brain overcoming the presence of blood–brain barrier (meninges) [8,9]. 6. Drug loading onto nanoparticles modifies cell and tissue distribution and leads to a more selective delivery of biologically active compounds to enhance drug efficacy and reduces drug toxicity [10,11].

## Applications of nanobiotechnology in medical and clinical fields

A number of clinical applications of nanobiotechnology, such as disease diagnosis, target-specific drug delivery, and molecular imaging are being laboriously investigated at present. Some new promising products are also undergoing clinical trials [12,13]. Such advanced applications of this approach to biological systems will undoubtedly transform the foundations of diagnosis, treatment, and prevention of disease in future. Some of these applications are discussed below.

(a) Diagnostic applicationsCurrent diagnostic methods for most diseases depend on the manifestation of visible symptoms before medical professionals can recognize that the patient suffers from a specific illness. But by the time those symptoms have appeared, treatment may have a decreased chance of being effective. Therefore the earlier a disease can be detected, the better the chance for a cure is. Optimally, diseases should be diagnosed and cured before symptoms even manifest themselves. Nucleic acid diagnostics will play a crucial role in that process, as they allow the detection of pathogens and diseases/diseased cells at such an early symptomless stage of disease progression that effective treatment is more feasible. Current technology, such as- polymerase chain reaction (PCR) leads toward such tests and devices, but nanotechnology is expanding the options currently available, which will result in greater sensitivity and far better efficiency and economy.

1. Detection:Many currently used/conventional clinical tests reveal the presence of a molecule or a disease causing organism by detecting the binding of a specific antibody to the disease-related target. Traditionally, such tests are performed by conjugating the antibodies with inorganic/organic dyes and visualizing the signals within the samples through fluorescence microscopy or electronic microscopy. However, dyes often limit the specificity and practicality of the detection methods. Nanobiotechnology offers a solution by using semiconductor nanocrystals (also referred to as "quantum dots"). These minuscule probes can withstand significantly more cycles of excitations and light emissions than typical organic molecules, which more readily decompose [14].

2. Individual target probesDespite the advantages of magnetic detections, optical and colorimetric detections will continue to be chosen by the medical community. Nanosphere (Northbrook, Illinois) is one of the companies that developed techniques that allow/allowing doctors to optically detect the genetic compositions of biological specimens. Nano gold particles studded with short segments of DNA form the basis of the easy-to-read test for the presence of any given genetic sequence. If the sequence of interest in the samples, it binds to complementary DNA tentacles on multiple nanospheres and forms a dense web of visible gold balls. This technology allows/facilitates the detection of pathogenic organisms and has shown promising results in the detection of anthrax, giving much higher sensitivity than tests that are currently being used [15].

3. Protein chipsProteins play the central role in establishing the biological phenotype of organisms in healthy and diseased states and are more indicative of functionality. Hence, proteomics is important in disease diagnostics and pharmaceutics, where drugs can be developed to alter signaling pathways. Protein chips can be treated with chemical groups, or small modular protein components, that can specifically bind to proteins containing a certain structural or biochemical motif [16]. Two companies currently operating in this application space are Agilent, Inc. and NanoInk, Inc. Agilent uses a non-contact ink-jet technology to produce microarrays by printing oligos and whole cDNAs onto glass slides at the nanoscale. NanoInk uses dip-pen nanolithography (DPN) technology to assemble structure on a nanoscale of measurement [17].

4. Sparse cell detectionSparse cells are both rare and physiologically distinct from their surrounding cells in normal physiological conditions (e.g. cancer cells, lymphocytes, fetal cells and HIV-infected T cells). They are significant in the detection and diagnosis of various genetic defects. However, it is a challenge to identify and subsequently isolate these sparse cells. Nanobiotechnology presents new opportunities for advancement in this area. Scientists developed nanosystems capable of effectively sorting sparse cells from blood and other tissues. This technology takes advantage of/exploits the unique properties of sparse cells manifested in differences in deformation, surface charges and affinity for specific receptors and/or ligands. For example, by inserting electrodes into microchannels, cells can be precisely sorted based on surface charge. They can also be sorted by using biocompatible surfaces with precise nanopores. The nano-biotechnology center at Cornell University (NBTC) is currently using these technologies to develop powerful diagnostic tools for the isolation and diagnosis of various diseases [18].

5. Nanotechnology as a tool in imagingIntracellular imaging can be made possible through labelling of target molecules with quantum dots (QDs) or synthetic chomophores, such as fluorescent proteins that will facilitate direct investigation of intracellular signalling complex by optical techniques, i. e. confocal fluorescence microscopy or correlation imaging [19,20].

(b) Therapeutic applications:Nanotechnology can provide new formulations of drugs with less side effects and routes for drug delivery.

1. Drug Delivery:Nanoparticles as therapeutics can be delivered to targeted sites, including locations that cannot be easily reached by standard drugs. For instance, if a therapeutic can be chemically attached to a nanoparticle, it can then be guided to the site of the disease or infection by radio or magnetic signals. These nanodrugs can also be designed to "release" only at times when specific molecules are present or when external triggers (such as infrared heat) are provided. At the same time, harmful side effects from potent medications can be avoided by reducing the effective dosage needed to treat the patient. By encapsulating drugs in nanosized materials (such as organic dendrimers, hollow polymer capsules, and nanoshells), release can be controlled much more precisely than ever before. Drugs are designed to carry a therapeutic payload (radiation, chemotherapy or gene therapy) as well as for imaging applications [21]. Many agents, which cannot be administered orally due to their poor bioavailability, will now have scope of use in therapy with the help of nanotechnology [22,23]. Nano-formulations offer protection for agents vulnerable to degradation or denaturation when exposed to extreme pH, and also prolong half-life of a drug by expanding retention of the formulation through bioadhesion [24,25]. Another broad application of nanotechnology is the delivery of antigens for vaccination [26,27]. Recent advances in encapsulation and development of suitable animal models have demonstrated that microparticles and nanoparticles are capable of enhancing immunization [28].

2. Gene deliveryCurrent gene therapy systems suffer from the inherent difficulties of effective pharmaceutical processing and development, and the chance of reversion of an engineered mutant to the wild type. Potential immunogenicity of viral vectors involved in gene delivery is also problematic [29,30]. To address this issue, nanotechnological tools in human gene therapy have been tested and nanoparticle-based nonviral vectors (usully 50-500 nm in size) in transportation of plasmid DNA described. Therefore, successful introduction of less immunogenic nanosize gene carriers as a substitution of the disputed viral vectors seems beneficial in repairing or replacing impaired genes in human [31].

3. LiposomesA liposome being composed of a lipid bilayer can be used in gene therapy due to its ability to pass through lipid bilayers and cell membranes of the target. Recent use of several groups of liposomes in a local delivery has been found to be convincingly effective [32,33]. Liposomes can also help achieve targeted therapy. Zhang *et al* demonstrated widespread reporter expression in the brains of rhesus monkeys by linking nanoparticle (such as polyethylene glycol) treated liposomes to a monoclonal antibody for human insulin reporter [34]. These successful trials reflect the future of targeted therapy and the importance of nanometer-sized constructs for the advancement of molecular medicine.

4. SurfacesIn nature, there are a multitude of examples of the complicated interactions between molecules and surfaces. For example, the interactions between blood cells and the brain or between fungal pathogens and infection sites rely on complex interplays between cells and surface characteristics. Nanofabrication unravels the complexity of these interactions by modifying surface characteristics with nanoscale resolutions, which can lead to hybrid biological systems. This hybrid material can be used to screen drugs, as sensors, or as medical devices and implants. Nanosystems, owned by the Irish drug company Elan, developed a polymer coating capable of changing the surface of drugs that have poor water solubility [35].

5. Biomolecular EngineeringThe expense and time involved in traditional biomolecule designing limit the availability of bioactive molecules. Nanoscale assembly and synthesis techniques provide an alternative to traditional methods. Improvements can be achieved due to the ability to carry out chemical and biological reactions on solid substrates, rather than through the traditional solution based processes. The use of solid substrate usually means less waste and the ability to manipulate the biomolecule far more precisely. EngeneOS (Waltham, Massachusetts) pioneered the field of biomolecular engineering. The company developed the engineered genomic operating systems that create programmable biomolecular machines employing natural and artificial building blocks. These biomolecule machines have broad range of commercial applications-as biosensors, in chemical synthesis and processing, as bioelectronic devices and materials, in nanotechnology, in functional genomics and in drug discovery.

6. BiopharmaceuticalsNanobiotechnology can develop drugs for diseases that conventional pharmaceuticals cannot target. The pharmaceutical industry traditionally focuses on developing drugs to treat a defined universe of about five hundred confirmed disease targets. But approximately 70 to 80 percent of the new candidates for drug development fail, and these failures are often discovered late in the development process, with the loss of millions of dollars in R&D investments. Nanoscale techniques for drug development will be a boon to small companies, which cannot employ hundreds of organic chemists to synthesize and test thousands of compounds. Nanobiotechnology brings the ability to physically manipulate targets, molecules and atoms on solid substrates by tethering them to biomembranes and controlling where and when chemical reactions take place, in a fast process that requires few materials (reagents and solutions). This advance will reduce drug discovery costs, will provide a large diversity of compounds, and will facilitate the development of highly specific drugs. Potentia Pharmaceuticals (Louisville, Kentucky) is an early-stage company that is attempting to streamline the drug development process with the use of nanotechnologies (Harvard Business School 2001).

7. Nanotechnology in cardiac therapyNanotechnology is currently offering promising tools for applications in modern cardiovascular science to explore existing frontiers at the cellular level and treat challenging cardiovascular diseases more effectively. These tools can be applied in diagnosis, imaging and tissue engineering [36]. Miniaturized nanoscale sensors like quantum dots (QDs), nanocrystals, and nanobarcodes are capable of sensing and monitoring complex immune signals in response to cardiac or inflammatory events [20]. Nanotechnology can also help detect and describe clinically-significant specific mechanisms implicated in cardiac disorders. In addition, it is useful in designing atomic-scale machines that can be incorporated into biological systems at the molecular level. Introduction of these newly designed nanomachines may positively change many ideas and hypotheses in the treatment of critical cardiovascular diseases. Nanotechnology could also have great impact in tackling issues like unstable plaques and clarification of valves. Thus, this approach could be a real milestone of success in achieving localized and sustained arterial and cardiac drug therapy for the management of cardiovascular diseases [37].

8. Nanotechnology in dental careNanotechnology will have future medical applications in the field of dentistry. The role of nanodentistry by means of the use of nanomaterials [38,39], biotechnology [40,41], and nanorobotics will ensure better oral health. Millions of people currently receiving poor dental care will benefit from such remarkable breakthrough in the science of dental health [42,43]. Moreover, nanodental techniques in major tooth repair may also evolve. Reconstructive dental nanorobots could be used in selective and precise occlusion of specific tubules within minutes, and this will facilitate quick and permanent recovery. The advantage of nanodentistry in natural tooth maintenance could also be significant [44]. Covalently-bonded artificial materials like sapphire may replace upper enamel layer to boost the appearance and durability of teeth [43].

9. Nanotechnology in orthopedic applicationsNanomaterials sized between 1 and 100 nm have role to play as new and functional constituents of bones being also made up of nanosized organic and mineral phases [45,46]. Nanomaterials, nanopolymers, carbon nanofibers, nanotubes, and ceramic nanocomposites may help with more efficient deposition of calcium-containing minerals on implants. Based on these evidences and observations, nanostructure materials represent a unique realm of research and development that may improve the attachment of an implant to the surrounding bone matters by enhancing bone cell interactions, and this will indeed aid in improving orthopedic implant efficacy while drastically minimizing patient-compliance problems.

## Future prospects of nanobiotechnology

There is much debate on the future implications of nanobiotechnology. It could create and suggest implementation of a choice of various new materials and devices potentially useful in the field of medicine, electronics, biomaterials and energy production. Nevertheless, this approach raises many of the same issues as any new technology, including problems with toxicity and environmental impact of nanomaterials [47] and their potential effects on global economics, as well as speculation about various doomsday scenarios. These concerns have accounted for a debate among advocacy groups and governments on whether special statutory regulation of nanobiotechnology is warranted.

Despite the existence of some disputes, this technology renders immense hope for the future. It may lead to innovations by playing a prominent role in various biomedical applications ranging from drug delivery and gene therapy to molecular imaging, biomarkers and biosensors. One of these applications being the prime research objective of the present time would be target-specific drug therapy and methods for early diagnosis and treatment of diseases [2]. Two types of medical applications are already emerging, both in clinical diagnosis and in R&D. Imaging applications, such as quantum dot technology are already being licensed and applications for monitoring cellular activities in tissue are coming soon. The second major type of application involves the development of highly specific and sensitive means of detecting nucleic acids and proteins [48]. By 2015 to 2020, we will see that products being tested in academic and government laboratories will be creeping into commercialization. Sparse cell isolation and molecular filtration applications should, by then, make it to market. Some of the drug delivery systems should be commercialized or in advanced clinical trials. For example - drug delivery systems have been developed by NanoSystems or by American Pharmaceutical Partners, which is testing the encapsulation of Taxol, a cancer drug in a nanopolymer called paclitaxel. Most medical devices and therapeutics are a decade or more away from market. Therefore, drug target manipulation as well as device implantation requires a complex technical infrastructure like nanotechnology as well as complex regulatory management [49].

Continuous advancements in nanomedicine have opened up its opportunities for application in a variety of medical disciplines. Its future application as diagnostic and regenerative medicine is currently being investigated. In diagnosis, detection of diseased cells would be faster, possibly at the point of a single sick cell, while allowing diseased cells to be cured at once before they spread into and affect other parts of the body. Also, individuals suffering from major traumatic injuries or impaired organ functions could benefit from the use of nanomedicine.

## Challenges for nanobiotechnology

No single person can provide the answers to challenges that nanotechnology brings, nor can any single group or intellectual discipline. The five main challenges are to develop instruments to assess exposure to engineered nano-materials in the air and water. It is fairly understood that exposure of humans and animals to the environment potentially contaminated with nano-materials may need to be monitored for any adverse consequence. The challenge becomes increasingly difficult in more complex matrices like food. The second challenge would be to develop applicable methods to detect and determine the toxicity of engineered nano-materials within next 5 to 15 years. Then again, proposing models for predicting effects of these nano-materials on human health and the environment would be an inevitable issue. The next challenge would be to develop reverse systems to evaluate precise impact of engineered nano-materials on health and the environment over the entire life span that speaks to the life cycle issue. The fifth being more of a grand challenge would be to develop the tools to properly assess risk to human health and to the environment. Commercialization challenges of nanobiotechnology include uncertainty of effectiveness of innovation, scalability, funding, scarce resources, patience etc. A broad majority of company recognizes a great potential in nanotechnology for the development of new products and the improvement of existing products. A new potentially disruptive technology like nanotechnology raises fundamental questions about the need for new regulations. Authorities around the world should evaluate possible risks and an appropriate regulatory response to the extensive use of this advanced technology.

## Potential hazards of nanoparticles

Nanoparticles, as a result of their extreme microscopic dimension, which gives unique advantage, have potential hazards similar to particulate matters [50]. These particles have the potential to cause varied pathologies of respiratory, cardiovascular and gastrointestinal system [51]. Intra-tracheal instillation of carbon nanotube particles in mice has shown that carbon nanotubes have the potential to cause varied lung pathologies like epitheloid granuloma, interstitial inflammation, peribronchial inflammation and necrosis of lung. The toxicity produced by carbon nanotube was found to be greater than that produced by carbon black and quartz [52].

It has been shown that nanomaterials can enter the human body through several ports. Accidental or involuntary contact during production or use is most likely to occur via the lungs, from which a rapid translocation is possible to other vital organs through the bloodstream. On the cellular level, an ability to act as a gene vector has been demonstrated for nanoparticles [53]. Nanoparticles can enter the central nervous system either directly through axons of olfactory pathway or through systemic circulation through the olfactory bulb [54]. Studies done on monkeys and rats have shown accumulation of carbon and manganese nanoparticles in the olfactory bulb through the olfactory pathway [55]. This shows that nanoparticle-mediated delivery can, in future, provide a means of alternate route, circumventing the blood brain barrier. However, this can also result in the inflammatory reactions/responses in the brain, which needs to be evaluated.

Radomski *et al*[56] have observed the pro-aggregatory effects of nanotubes on platelets in *in vitro* studies and acceleration of vascular thrombosis in rat. It was also observed that fullerenes do not have the property of inducing platelet aggregation. Thus, for designing nanoparticle-based drug delivery systems, fullerenes may be a safer approach as compared to nanotubes [57].

The toxicity of nanoparticles can also be extrapolated to gastrointestinal system, resulting in inflammatory bowel diseases. The toxicity of nanoparticles may be related to its ability to induce release of pro-inflammatory mediators resulting in inflammatory response and organ damage. If ingested, the nanoparticles can reach the circulation and reach different organs and systems and possibly result in toxicity [58]. These have been studied *in vitro* and in animal models and the effect on human system is difficult to extrapolate from such studies. Their use in humans requires further research and much needed caution.

## Conclusion

Nanobiotechnology is still in its early stages. The multidisciplinary field of nanobiotechnology is bringing the science of the almost incomprehensibly small device closer and closer to reality. The effects of these developments will at some point be so vast that they will probably affect virtually all fields of science and technology. Nanobiotechnology offers a wide range of uses in medicine. Innovations such as drug delivery systems are only the beginnings of the start of something new. Many diseases that do not have cures today may be cured by nanotechnology in the future. Although the expectations from nanobiotechnology in medicine are high and the potential benefits are endlessly enlisted, the safety of nanomedicine is not yet fully defined. Use of nanotechnology in medical therapeutics needs adequate evaluation of its risk and safety factors. Scientists who are against the use of nanotechnology also agree that advancement in nanotechnology should continue because this field promises great benefits, but testing should be carried out to ensure the safety of the people. It is possible that nanomedicine in future would play a crucial/unparallel role in treatment of human diseases and also in enhancement of normal human physiology. If everything runs smoothly, nanobiotechnology will, one day, become an inevitable part of our everyday life and will help save many lives.

## Competing interests

The authors declare that they have no competing interests.

## Authors' contributions

MF planned the study and outlined it, prepared final manuscript. ZH performed literature review and helped in preparing manuscript. HA also performed literature review and helped in preparing manuscript. All authors read and approved the final manuscript.

## References

[B1] EmerichDFThanosCGNanotechnology and medicineExpert Opin Biol Ther2003365566310.1517/14712598.3.4.65512831370

[B2] SahooKSLabhasetwarVNanotech approaches to drug delivery and imagingDDT2003824111211201467873710.1016/s1359-6446(03)02903-9

[B3] VasirJKLabhasetwarVTargeted drug delivery in cancer therapyTechnol Cancer Res Treat200543633741602905610.1177/153303460500400405

[B4] VasirJKReddyMKLabhasetwarVNanosystems in drug targeting: opportunities and challengesCurr Nanosci20051476410.2174/1573413052953110

[B5] MaedaHWuJSawaTMatsumuraYHoriKTumor vascular permeability and the EPR effect in macromolecular therapeutics: a reviewJ Control Release20006527128410.1016/S0168-3659(99)00248-510699287

[B6] MatsumuraYMaedaHA new concept for macromolecular therapeutics in cancer chemotherapy: mechanism of tumoritropic accumulation of proteins and the antitumor agent smancsCancer Res198646638763922946403

[B7] AllenTMCullisPRDrug delivery systems: entering the mainstreamScience20043031818182210.1126/science.109583315031496

[B8] AlyautdinRNTezikovEBRamgePKharkevichDABegleyDJKreuterJSignificant entry of tubocurarine into the brain of rats by adsorption to polysorbate 80-coated polybutylcyanoacrylate nanoparticles: an in situ brain perfusion studyJ Microencapsul199815677410.3109/026520498090068369463808

[B9] Garcia-GarciaEGilSAndrieuxKDesmaëleDNicolasVTaranFGeorginDAndreuxJPRouxFCouvreurPA relevant in vitro rat model for the evaluation of blood–brain barrier translocation of nanoparticlesCell Mol Life Sci200562121400140810.1007/s00018-005-5094-315905957PMC2773840

[B10] FengSSMuLWinKYNanoparticles of biodegradable polymers for clinical administration of paclitaxelCurr Med Chem20041141342410.2174/092986704345590914965222

[B11] de KozakYAndrieuxKVillarroyaHKleinCThillaye-GoldenbergBNaudMCIntraocular injection of tamoxifen-loaded nanoparticles: a new treatment of experimental autoimmune uveoretinitisEur J Immunol2004343702371210.1002/eji.20042502215517615

[B12] ShafferCNanomedicine transforms drug deliveryDrug Discov Today200510158115821637681010.1016/S1359-6446(05)03654-8

[B13] MoghimiSMHunterACMurrayJCNanomedicine: current status and future prospectsFASEB J20051931133010.1096/fj.04-2747rev15746175

[B14] DrexlerEKNanosytems: Molecular Machinery, Manufacturing and Computation1992John Wiley & Sons, New York

[B15] Nanosphere Inc2004Available at http://www.nanosphere-inc.com

[B16] LeeKBParkSJMirkinCSmithJMrKischMAProtein Nanoarrays generated by Dip-Pen NanolithographyScience20022951702170510.1126/science.106717211834780

[B17] NanoInk Inc2004Available at http://www.nanoink.net

[B18] NBTC (Nano-biotechnology Center, Cornell University)2004Available at http://www.nbtc.cornell.edu/default.htm

[B19] LinHDatarRHMedical applications of nanotechnologyNatl Med J India200619273216570683

[B20] GuccioneSLiKCBednarskiMDVascular-targeted nanoparticles for molecular imaging and therapyMethods Enzymol20043862192361512025410.1016/S0076-6879(04)86010-5

[B21] LaVanDALynnDMLangerRTimeline: Moving Smaller in drug discovery and deliveryNat Rev Drug Discov20021778410.1038/nrd70712119612

[B22] El-ShabouriMHPositively charged nanoparticles for improving the oral bioavailability of cyclosporin-AInt J Pharm200224910111810.1016/S0378-5173(02)00461-112433438

[B23] HuLTangXCuiFSolid lipid nanoparticles (SLNs) to improve oral bioavailability of poorly soluble drugsJ Pharm Pharmacol200456152715351556375910.1211/0022357044959

[B24] ArangoaMACampaneroMARenedoMJPonchelGIracheJMGliadin nanoparticles as carriers for the oral administration of lipophilic drugs. Relationships between bioadhesion and pharmacokineticsPharm Res2001181521152710.1023/A:101301811182911758758

[B25] ArbosPCampaneroMAArangoaMAIracheJMNanoparticles with specific bioadhesive properties to circumvent the pre-systemic degradation of fluorinated pyrimidinesJ Control Release200496556510.1016/j.jconrel.2004.01.00615063029

[B26] DiwanMElamanchiliPLaneHGainerASamuelJBiodegradable nanoparticle mediated antigen delivery to human cord blood derived dendritic cells for induction of primary T cell responsesJ Drug Target20031149550710.1080/1061186041000167002615203918

[B27] Koping-HoggardMSanchezAAlonsoMJNanoparticles as carriers for nasal vaccine deliveryExpert Rev Vaccines2005418519610.1586/14760584.4.2.18515889992

[B28] LutsiakMERobinsonDRCoesterCKwonGSSamuelJAnalysis of poly (d, l-lactic-co-glycolic acid) nanosphere uptake by human dendritic cells and macrophages in vitroPharm Res2002191480148710.1023/A:102045253182812425465

[B29] YotsuyanagiTHazemotoNCationic liposomes in gene deliveryNippon Rinsho1998567057129549361

[B30] YoungLSSearlePFOnionDMautnerVViral gene therapy strategies: from basic science to clinical applicationJ Pathol200620829931810.1002/path.189616362990

[B31] DavisSSBiomedical applications of nanotechnology—implications for drug targeting and gene therapyTrends Biotechnol19971521722410.1016/S0167-7799(97)01036-69183864

[B32] HartSLLipid carriers for gene therapyCurr Drug Deliv2005242342810.2174/15672010577437023016305445

[B33] EwertKEvansHMAhmadASlackNLLinAJMartin-HerranzALipoplex structures and their distinct cellular pathwaysAdv Genet20055311915516240992

[B34] ZhangYSchlachetzkiFLiJYBoadoRJPardridgeWMOrgan specific gene expression in the rhesus monkey eye following intravenous nonviral gene transferMol Vis2003946547214551536

[B35] Elan Corporation, PLC2004Available at http://www.elan.com

[B36] WicklineSANeubauerAMWinterPCaruthersSLanzaGApplications of nanotechnology to atherosclerosis, thrombosis, and vascular biologyArterioscler Thromb Vasc Biol2006264354411637360910.1161/01.ATV.0000201069.47550.8b

[B37] PanyamJLabhasetwarVBiodegradable nanoparticles for drug and gene delivery to cells and tissueAdv Drug Deliv Rev20035532934710.1016/S0169-409X(02)00228-412628320

[B38] WestJLHalasNJApplications of nanotechnology to biotechnology commentaryCurr Opin Biotechnol20001121521710.1016/S0958-1669(00)00082-310753774

[B39] ShiHTsaiWBGarrisonMDFerrariSRatnerBDTemplateimprinted nanostructured surfaces for protein recognitionNature199939859359710.1038/1926710217142

[B40] SimsMRBrackets, epitopes and flash memory cards: a futuristic view of clinical orthodonticsAust Orthod J19991526026810806932

[B41] SlavkinHCEntering the era of molecular dentistryJ Am Dent Assoc19991304134171008566510.14219/jada.archive.1999.0212

[B42] UreDHarrisJNanotechnology in dentistry: reduction to practiceDent Update20033010151261930710.12968/denu.2003.30.1.10

[B43] FartashBTangerudTSilnessJArvidsonKRehabilitation of mandibular edentulism by single crystal sapphire implants and overdentures: 3-12 year results in 86 patients. A dual center international studyClin Oral Implants Res1996722022910.1034/j.1600-0501.1996.070304.x9151586

[B44] ShellhartWCOesterleLJUprighting molars without extrusionJ Am Dent Assoc19991303813851008566110.14219/jada.archive.1999.0208

[B45] WebsterTJWaidMCMcKenzieJLPriceRLEjioforJUNanobiotechnology: carbon nanofibres as improved neural and orthopedic implantsNanotechnology200415485410.1088/0957-4484/15/1/00934911207

[B46] PriceRLWaidMCHaberstrohKMWebsterTJSelective bone cell adhesion on formulations containing carbon nanofibersBiomaterials2003241877188710.1016/S0142-9612(02)00609-912615478

[B47] BuzeaCPachecoIRobbieKNanomaterials and nanoparticles: Sources and ToxicityBiointerphases20072MR1710.1116/1.281569020419892

[B48] MilunovichSRoyJThe next small thing: An Introduction to nanotechnology. Merrill Lynch Report, September 4, 2001

[B49] Hamad-SchifferliKSchwartzJSantosATZhangSJacobsonJRemote electronic control of DNA hybridization through inductive coupling to an attached metal nanocrystal antennaNature200241515215510.1038/415152a11805829

[B50] LiZHuldermanTSalmenRChapmanRLeonardSSYoungSHCardiovascular effects of pulmonary exposure to single-wall carbon nanotubesEnviron Health Perspect20071153773821743148610.1289/ehp.9688PMC1849906

[B51] NijharaRBalakrishnanKBringing nanomedicines to market: regulatory challenges, opportunities, and uncertaintiesNanomedicine2006212713610.1016/j.nano.2006.04.00517292125

[B52] LamCWJamesJTMcCluskeyRHunterRLPulmonary toxicity of single-wall carbon nanotubes in mice 7 and 90 days after intratracheal instillationToxicol Sci2004771261341451495810.1093/toxsci/kfg243

[B53] WilliamsDThe risks of nanotechnologyMed Device Technol20041591016438441

[B54] OberdorsterEManufactured nanomaterials (fullerenes, C60) induce oxidative stress in the brain of juvenile largemouth bassEnviron Health Perspect20041121058106210.1289/ehp.702115238277PMC1247377

[B55] ElderAGeleinRSilvaVFeikertTOpanashukLCarterJTranslocation of inhaled ultrafine manganese oxide particles to the central nervous systemEnviron Health Perspect20061141172117810.1289/ehp.903016882521PMC1552007

[B56] RadomskiAJuraszPOnso-EscolanoDDrewsMMorandiMMalinskiTNanoparticle-induced platelet aggregation and vascular thrombosisBr J Pharmacol200514688289310.1038/sj.bjp.070638616158070PMC1751219

[B57] MedinaCSantos-MartinezMJRadomskiACorriganOIRadomskiMWNanoparticles : pharmacological and toxicological significanceBr J Pharmacol20071505525581724536610.1038/sj.bjp.0707130PMC2189773

[B58] ChenZMengHXingGChenCZhaoYJiaGAcute toxicological effects of copper nanoparticles in vivoToxicol Lett200616310912010.1016/j.toxlet.2005.10.00316289865

